# Auricular Point Acupressure Combined with Compound Lidocaine Cream to Manage Arteriovenous Fistula Puncture Pain: A Multicenter Randomized Controlled Trial

**DOI:** 10.1155/2021/5573567

**Published:** 2021-07-28

**Authors:** Xiaohui Liu, Wei Wei, Yaqi Wu, Xiao Jiang, Xueqin Liu, Ying Zhang, Chao Hsing Yeh, Yuejuan Zhang

**Affiliations:** ^1^Department of Nursing, The First Affiliated Hospital of Hunan University of Chinese Medicine, Changsha, Hunan 410007, China; ^2^Department of Traditional Chinese Medicine Nursing, Nursing College of Henan University of Traditional Chinese Medicine, Zhengzhou, Henan 473005, China; ^3^College of Nursing, Henan University of Traditional Chinese Medicine, Zhengzhou, Henan 473005, China; ^4^Johns Hopkins University School of Nursing, 525 N. Wolfe Street, Room 421, Baltimore, MD 21205, USA

## Abstract

**Background:**

Arteriovenous fistula (AVF) puncture pain is an inevitable problem for maintenance hemodialysis (MHD) patients and may seriously endanger the physical and mental health of patients with MHD. Studies have shown that drug or nondrug measures can reduce AVF puncture pain, but much improvement is needed. When combined with compound lidocaine cream (CLC) in the treatment of AVF puncture pain, auricular point acupressure (APA)—a therapeutic method in which specific points on the auricle of the outer ear are stimulated to treat various disorders of the body—and the therapeutic value and synergistic effects of auriculotherapy merit further investigation.

**Methods:**

120 MHD patients were recruited at blood purification centers in three hospitals between January 2016 and April 2019. After completion of the baseline survey, all patients were randomly divided by the envelope method into a control group, APA group, CLC group, and APA combined with CLC, with 30 subjects per group. The numerical rating scale (NRS) of pain was used to measure the pain before intervention and 1, 4, and 8 weeks after intervention. The State-Trait Anxiety Inventory (STAI), General Comfort Questionnaire (GCQ), blood pressure, and heart rates were obtained before and after the intervention.

**Results:**

Pain, anxiety, comfort, blood pressure (BP), and heart rates (HR) of the three groups were better than those of the control group; the difference was statistically significant (*P* < 0.05). In addition, the APA combined with CLC group was better than the APA group and CLC group, respectively, in those outcomes (*P* < 0.05).

**Conclusion:**

Both APA and CLC can effectively relieve AVF puncture pain, and the combined application has more outstanding effects.

## 1. Introduction

As aging society intensifies, the incidence rate of end-stage renal disease (ESRD) increases due to the high prevalence of hypertension and diabetes that causes the end stage of irreversible renal failure [1]. China has the largest number of ESRD patients in the world; in 2020, an estimated two million people suffered from ESRD [2]. ESRD has become a serious worldwide public health problem [3]. But the life expectancy of ESRD patients has been greatly prolonged because of hemodialysis (HD), which can remove wastes and fluid from blood [4].

HD is a procedure that involves diverting blood into an external machine to filter the blood to remove the waste and extra fluid before the blood returns back to the body. HD includes three sessions a week, and each session lasts around 4 hours using a blood vessel with an arteriovenous fistula (AVF) [5]. For the sake of dialysis adequacy, two 16-18G puncture needles are required to insert AVF for each HD treatment, which means that patients with maintenance hemodialysis (MHD) need to endure more than 300 AVF punctures each year [6, 7]. While continuing their lives, patients suffer from pain and strain on the AVF puncture sites. Although the long-term AVF puncture pain is considered a necessary part of the HD procedure [8, 9], the AVF puncture pain imposes a series of harmful effects on HD patients, including stress-induced high blood pressure and fast heart rates [10]. Psychologically, AVF puncture pain causes pressure, tension, anxiety, depression, and fear [9]. Moreover, the greater the AVF puncture pain, the lower quality of life for MHD patients [1, 11].

The literature shows that lidocaine preparations and several non-drug measures have positive effects to alleviate AVF puncture pain, including lidocaine formulations that include lidocaine cream [12], lidocaine spray [13], or nanoemulsion [14]. Complementary and alternative medicine (CAM) approaches have been shown to enhance pain relief, including music therapy [7], aromatherapy [10], Rose fixed oil [15], cryotherapy [9], moxibustion [16], herb (*Fumaria parviflora* L. [17]), and relaxation training [18]. Chronic pain impacts not only physical function, but also psychophysiological and social domains; thus, ideal pain management indicates that multimodal analgesia and preemptive analgesia have better outcomes [19, 20]. Lidocaine cream is a commonly used lidocaine preparation that is easy to use and acquire. However, other treatment modalities, such as musical therapy or aromatherapy, are not practical for MHD patients in China due to the limited space during HD procedures. Relaxation training requires professional psychological training, which is not a common practice in China yet. Therefore, additional nonpharmacological strategies are needed to enhance the pain relief for MHD patients.

Auricular point acupressure (APA) is a branch of acupuncture and moxibustion in Traditional Chinese Medicine (TCM). APA—using plant seeds or magnetic beads to press the acupoints on the ear for disease prevention and treatment—is included in routine nursing practice in China [21, 22]. Human beings have used auricular therapy to treat diseases for more than 3,000 years [23]. The mechanism of APA includes meridians, nerves, and somatic reflex [24]. APA can be performed by nurses who first tape seeds/or magnetics on the patients ear acupoints with tape; then patients continue to press the seeds/magnetics on their ears to achieve therapeutic effects. It is a noninvasive and self-management technique for patients to manage their pain. Clinical studies have shown that APA can relieve chronic neck pain [25], chronic low back pain [26], acute postoperative pain [27], labor pain [28], and AVF puncture pain [29]. Liu et al. designed a control group to determine the efficacy of APA to manage AVF puncture pain in HD patients [29]. However, its evidence-based quality is low. Thus, the purpose of this study was to evaluate the effectiveness of the APA combined with lidocaine in the treatment of AVF puncture pain.

## 2. Materials and Methods

### 2.1. Study Design, Setting, and Ethics

This was a prospective, parallel-group, single-blind, randomized trial conducted in 128 adult patients aged 18–78 years diagnosed with MHD patients with AVF puncture at Henan Province Hospital of Traditional Chinese medicine. The study protocol and informed consent forms were reviewed and approved by the Institutional Review Board of Henan Province Hospital of Traditional Chinese medicine (the second affiliated hospital of Henan University of Traditional Chinese Medicine) at Zhengzhou on November 11, 2016 (Ethical code: 2016111501).

During the screening visit, information regarding demographic characteristics, medical history, and arteriovenous fistula was collected after the signed informed consent form was obtained from the participants. The eligible participants were randomly allocated to the following groups: (1) Compound Lidocaine Cream (CLC), (2) Auricular point acupressure (APA), (3) CLC + APA, and (4) control (usual care). The participants were administered corresponding protocol for 8 consecutive weeks, respectively. For screening assessments, the validated self-reported outcomes for pain were used to measure before intervention and 1, 4 and, 8 weeks after intervention. The second outcomes such as anxiety intensity, comfort severity, blood pressure, and heart rates were evaluated at baseline and the endpoint. The safety of the APA and CLC was assessed by performing the local skin condition and adverse event reporting.

### 2.2. Participants

Inclusion criteria were as follows: (1) patients were18 years of age or older; (2) they had undergone three sessions of HD/week for MHD patients with AVF puncture for at least 3 months; (3) patients with puncture pain average scores ≥ 4 were screened on an 11-point numerical pain scale for in-the-past three administrations of AVF fistula punctures.

Exclusion criteria were as follows: (1) unable to cooperate with study activities due to critical condition; (2) skin damage, scar, or skin allergy at the puncture site or ear skins; (3) history of allergic reactions to experimental drug (Lidocaine). Exit criteria were as follows: during the study period, some patients died due to disease, treatment changes, or drug reactions, and renal transplant treatment patients could not continue to participate in the study or were actively asked to withdraw.

### 2.3. Randomization and Allocation Concealment

The determination of sample size was based on experimental purposes of the study and experience. We generated random numbers online (https://www.random.org). The three centers put the random numbers into a uniform and opaque envelope; the envelopes were kept out of the reach of patients in each center. After confirming that a patient met the inclusion criteria, a random number was drawn by the patient, and the random number obtained by the patient was divided by 4. Being divisible by 4 was assigned to the control group, the remaining 1 was assigned to the CLC group, the remaining 2 were assigned to the APA group, and the remaining 3 were assigned to the CLC + APA group.

### 2.4. Sample Size

In total, 128 eligible participants were randomly divided into the control group (A group, *n* = 32), the CLC group (B group, *n* = 32), the APA group (C group, *n* = 32), or the CLC + APA group (D group), *n* = 32) (Figure 1). During the intervention, eight participants changed their HD process and were thus eliminated by the study team (2 participants in each group). A total of 120 participants who completed all data collection were included in the final analysis.

### 2.5. HD Routine Procedures

All participating patients received the same HD protocol (i.e., 3 sessions of HD/week, which lasted four hours each time for each session, anti-hypertensive drugs, erythropoietin, or heparin). The AVF punctures during the intervention were performed by four certified HD nurse specialists at each study setting. The nurses had more than five years of HD experience and regularly had at least 98% average success rates of AVF puncture at quarterly assessments. They were responsible for AVF puncture of the four groups of patients. All patients were punctured with a standard rope ladder. The needle was inserted at an angle of more than 40° and the needle tip inclined upward. The arterial puncture needle was punctured in the distal direction, and the venous puncture needle was punctured along the blood flow direction, while trying to avoid the influence of human factors on pain. A Japan Toray tr-8000 dialyzer was used for HD. Bipolar reverse osmosis water was used as a dialyzer. All patients were treated with a disposable rotary needle with a hole of 16 g (produced by Dalian Medical JMS Equipment Co., Ltd., 20143152113, Dalian, China).

### 2.6. Intervention

The 8-week intervention included the following four study groups.

#### 2.6.1. CLC Group

Participants enrolled in this group received CLC treatment (compound lidocaine cream; each Gram contained 25 mg of procaine and 25 mg of lidocaine; Tongfang Pharmaceutical Group Co., Ltd., Beijing, China, approval Number: gyzzh20063466). The CLC was applied to the puncture sites of AVF 60 min before HD with a dosage needle with a diameter of about 5 cm and a thickness of 2 cm on the skin and covered with preservative film. The local skin was cleaned before each puncture, and then the operation was carried out according to the routine puncture process.

#### 2.6.2. APA Group

Participants enrolled in this group received two APA treatments a week. Auricular points on the ears were detected with an electrical acupoint finder, which measures auricular cutaneous resistance to identify the potential acupoints for treatment. The Chinese Standard Ear Acupoint Chart, which is recognized by the World Health Organization [30], and the latest nomenclature and location of auricular points announced by the China Standardization Organizing Committee in 2008 (GB/T 13734-2008) were used as a guide to locate the active ear points for AVF puncture pain. According to Huang [31], the auricular treatment medicine, syndrome differentiation, and selection based on TCM renal disease and AVF puncture pain, nine auricular acupoints were selected: five points for alleviating stress and pain (i.e., shenmen [TF4], sympathetic point [AH6a], adrenal gland [TG2], endocrine [CO18], and nervous subcortex [AT4]), two corresponding to the anatomical location of the puncture sites (i.e., elbow [SF3] and wrist [SF2]), and three acupoints related to viscera function (i.e., heart [CO15], liver [CO12], and kidney [CO10]) (Figure 2). The acupoints can be stimulated at any order. Participants were instructed to evenly press (5 seconds) each taped beads covering each ear acupoint without rubbing (to avoid skin damage or movement of the seed from the ear point). A 2-second pause occurs between the pressings. All acupoints were affixed by the first author (Liu). After the acupoints were identified by the electrical finder, they were disinfected using the 75% alcohol, and the magnetic beads were clipped with tweezers and pasted on the selected acupoints of one ear and changed to the contralateral ear after 3 days of treatment. After tape placement, the first author demonstrated the pressing technique to the participants, instructing them to apply steady pressure on the taped seeds until either mild discomfort or tingling was felt. The stimulation was done by the participant by pressing the magnetics three minutes for all of the ear acupoints for AVF puncture including (1) 30 minutes before each AVF punctl the acupoints; (2) 3 minutes before the puncture: this was done by the nurse to press the magnetic bead with the thumb and index finger pressing method about 2-3 minutes until there was slight distending pain and fever on the ear; and (3) continuous stimulation during the puncture: the nurse continued to stimulate the ear acupoints and stopped pressing after the puncture was successful. The degree of puncture pain was assessed and recorded immediately. In addition, during the eight-week intervention period, participants were told to press the seeds three times per day (i.e., morning, noon, and evening) for 3 minutes each time (i.e., 9 minutes total). Participants were instructed to remove the tape and magnets from one ear after 3 days, so that the ear was free of tape/magnets for 3 days each time. This minimized the risk of an allergic reaction to the tape and allowed the acupoints to recover and restore sensitivity prior to the next treatment.

Participants in the other group, who were blinded to this assignment, were provided the opportunity to receive APA treatment after completing all assessments. APA used the same batch of Hwato magnetic beads by Suzhou Medical Supplies Factory Co., Ltd. Suzhou, China (Registration Certificate No.: sxzz 20162261231; Executive Standard No.: yzb/su0903-2013).

#### 2.6.3. CLC + APA Group

Participants enrolled in this group received CLC at 60 minutes and APA at 30 minutes before AVF puncture. The intervention procedures were the same as the CLC or APA group.

#### 2.6.4. Control Group

Participants enrolled in this group received routine care as described in the “HD Routine Procedures.”

### 2.7. Measurements

#### 2.7.1. Pain Intensity

The numerical rating scale (NRS) of pain intensity is a 10 cm long line with 10 scales on the back and is marked with “0” and “10” on both sides of the front; 0 represents no pain, and 10 represents the most severe pain. In this study, the side with the scale should be positioned with its back toward the patient, and the patient should mark the corresponding position of pain on it; the pain score was then evaluated according to its position. NRS is simple, rapid, accurate, and easy to operate. It has been widely used in clinical practice, and its reliability and validity have been confirmed by many studies [7]. In this study, the NRS was used to evaluate AVF puncture pain intensity and was measured at 5–10 min after AVF punctures were performed.

#### 2.7.2. State-Trait Anxiety Inventory (STAI)

STAI was composed of 40 items including instructions and two subscales [32]. Items 1–20 were the State Anxiety Scale (SAI); items 21–40 were the Trait Anxiety Scale (TAI). The scales reflected the patients' degree of state and trait anxiety [33]. The STAI was translated into Chinese in 1988, and the translation retest reliability SAI was 0.88, TAI was 0.90, and reliability and validity were satisfactory [32]. In this study, the SAI was used to evaluate the anxiety level of MHD patients with AVF puncture stress; the TAI was used to evaluate the anxiety level of MHD patients with AVF in peacetime. The scale was measured at baseline and postintervention.

#### 2.7.3. General Comfort Questionnaire (GCQ)

The Chinese version of the GCQ, revised by Zhao TL [34], was used to measure comfort. The scale included four dimensions: physical comfort (8 items), psychological comfort (9 items), social comfort (7 items), and environmental comfort (4 items). Taking the 1–4 points Likert scoring method, the higher the score, the more comfortable. The scale had good reliability, validity, and feasibility, the overall Cronbach's *α* coefficient was 0.935, and the *α* coefficient of each dimension was 0.879–0.930; the overall retest reliability correlation coefficient was 0.944, and the retest reliability correlation coefficient of each dimension is 0.817–0.924; the average content validity index of all items of the scale is 0.883 [34]. The scale was used to evaluate the comfort of MHD patients and measured before and after each intervention.

#### 2.7.4. Blood Pressure (BP) and Heart Rate (HR)

The BP (systolic and diastolic blood pressure) and HR before and after AVF puncture were measured to evaluate the changes of physiological indexes and the effect of the interventions.

#### 2.7.5. Demographics Survey

The survey was used to collect the general demographic and disease-related data of the study participants, including age, gender, educational background, marital status, religion, smoking, and working conditions.

### 2.8. Statistical Analysis

Descriptive statistics (frequency and constituent ratio) were used to describe the counting data, and the mean ± standard deviation ($\bar{x}\pm s$) was used to describe the measurement data. *T* tests, chi square tests, and one-way ANOVA were used to compare the differences between groups. A least significant difference test (LSD) was used for pairwise comparison. Cohen's d (*η*2) was used to estimate effect size. The inspection level was *α* = 0.05. IBM SPSS22.0 software was used to input and analyze the experimental data of this study.

## 3. Results

### 3.1. Characteristics of the Participants

Table 1 lists the demographics characteristics of the study participants. The MHD patients included in this study were between 18 and 78 years old, with an average age of (51.52 ± 14.43) years. The majority of the study participants were male (66%), half of them were married (57%), 48% had at least a high school or college education, 53% were not working, 23% had religious beliefs, and 43% of them smoked. The average monthly family income was between ¥2000 and ¥5000, accounting for 48% that represented middle-incomers.  Table 2 presents the comparison of the clinical characteristics of the study participants. Diabetes was the relatively more common primary disease for HD, accounting for 35%, with the dialysis experiences between 1 and 3 years (33%). Approximately 48% of patients had a complication (such as renal anemia, renal dystrophy, renal hypertension, and disorder of calcium and phosphorus metabolism).

### 3.2. Pain Intensity

Pain intensity was measured at four time points: before intervention, 1 week and 4 weeks after first intervention, and postintervention (Table 3).  Figure 3 shows the change pattern of pain intensity in the four groups. There was no significant difference in the NRS score between the four groups before intervention (*P* > 0.05); there was significant difference in NRS pain score between the four groups after intervention (*P* < 0.01, *η*^2^ = 0.521). Compared with the control group, the other three groups (CLC, APA, CLC + APA) had statistically significant differences in pain scores (*P* < 0.01). The CLC + APA group was better than groups CLC and APA in that the difference was statistically significant (*F* = 67.843, *P* < 0.001) (Table 3).

### 3.3. Anxiety

According to the results of the state and trait anxiety, there was no significant difference between the four groups before intervention (*P* > 0.05); there was significant difference between the four groups after intervention (*P* < 0.001, *η*^2^ = 0.232 for state anxiety and *η*^2^ = 0.365 for trait anxiety) (Table 4). Compared with group A, the overall scores of state and trait anxiety in the other three groups were statistically significant (*P* < 0.01), while the effect of the CLC + APA group was better than that of the APA and CLC (*P* < 0.05) groups.

### 3.4. Comfort

The one-way analysis of variance (ANOVA) revealed no significant difference with the four dimensions of physiological comfort, psychological comfort, social comfort, environmental comfort, and overall comfort scores among the four groups before the intervention (*P* > 0.05) (Table 5). After the intervention, except for the social comfort dimension, the other four dimensions of physical comfort, psychological comfort, environmental comfort, and overall comfort score were statistically significant (*P* < 0.05). After least significant difference pairwise comparison, the results showed that the difference between group A and the other groups was statistically significant; while the effect of the CLC + APA group was better than that of the CLC and APA groups, the difference was statistically significant (*P* < 0.05) (Table 5).

### 3.5. BP and HR

Table 6 shows that no significant differences were observed between the groups for BP and HR before the intervention (*P* > 0.05). After intervention, the BP and HR of the four groups were significantly different (*P* < 0.05). Compared with group A, the differences of BP and HR in the other three groups were statistically significant (*P* < 0.01); the effect of regulating systolic and diastolic blood pressure in the CLC + APA and APA groups was better than that in groups A and CLC (*P* < 0.01) (Table 6).

### 3.6. Safety Assessment

During the intervention, there was no allergic reaction to local anesthetics or ear tape, no pallor, erythema, edema, papules, watery spots or erosion in the local skin, and no burning, tingling, or other feeling in the local part of the patient, about which the patient was asked; no systemic adverse reactions were observed, and no other discomfort symptoms were observed.

## 4. Discussion

To the best of our knowledge, this is the first multicenter study of APA combined with lidocaine cream in the treatment of AVF puncture pain. Our results show that, with the increase of intervention time, the pain scores of three intervention groups decreased gradually at 1, 4, and 8 weeks after intervention. The average pain scores for the intervention groups (i.e., APA, CLC, CLC + APA) had fewer than 4 points; the average pain intensity in the control group was 5.48 points. Our results also show that the intervention taken in this study was effective. In addition, the effect of combined application was better than that of a noncombined application.

We also evaluated BP and HR, which objectively reflected the pain. It is worth noting that APA can stabilize BP and HR, which is consistent with previous studies [10]. We believe that pain relief is part of the reason why APA stabilizes BP and HR and is also related to the mechanism of APA [35]. Acupoints are selected for analgesia, such as Shenmen, subcortical, and endocrine. According to TCM, Shenmen has analgesic, sedative, and sedative effects and is an important point for pain relief. Sympathetic excitation has the function of regulating autonomic nerves, regulating meridians, and regulating qi, activating blood circulation and relieving pain; the Subcortex is the key point for regulating cortical excitation and inhibition, which has good analgesic effect. The combination of these acupoints can adjust the pain areas of the central nervous system and achieve the effect of sedation, spasmolysis, and pain relief.

We believe that the application of CLC and APA before puncture can reduce the fear of pain and increase the pain self-management. In addition, the stimulation in the process of APA distracts the attention of patients and reduces the negative emotions during the waiting period of pain. The psychological support of nurses after puncture is also helpful for patients' emotional catharsis, thus blocking the occurrence and transmission of pain information before, during, and after puncture, blocking the reaction link of body stress process, so as to reduce the degree of pain. It also suggested that multimodal analgesia in the CLC + APA group was beneficial to the maximization and integration of pain control.

### 4.1. Our Study Shows That APA with CLC Can Enhance the Pain Management Model in AVF Puncture Pain

With the development of medical technology, the life cycle of MHD patients has been prolonged, and symptom management is particularly important. Even if AVF is unobstructed and well positioned, puncture pain is the main symptom of AVF patients. Preemptive analgesia prevents central hyperactivity by blocking the afferent pathway at the injured site of the central nervous system, which is often used as part of multimodal analgesia [20]. Studies have shown the effectiveness of preemptive analgesia [36]. The application of APA or CLC before AVF puncture was consistent with the concept of preemptive analgesia. Moreover, the combination of the two belongs to multimodal analgesia, which is in line with the current pain management concept and provides a new idea for clinical AVF puncture pain management.

### 4.2. APA Combined with CLC Is Helpful in Relieving AVF Puncture Anxiety

Research shows that pain is closely related to anxiety, which is a common negative emotion of MHD patients [37]. As a strong stressor, AVF puncture leads to excessive stress response and enhanced pain. Tolerance to the limit can cause and aggravate emotional disorders and can form a vicious circle state, affecting the physical and mental health of patients. In this study, the anxiety level of patients was generally higher than that of normal patients [32], which means that patients were in a high stress state. The results showed that the anxiety degree of CLC, C, and D decreased significantly after intervention, and the difference was statistically significant compared with the control group, but the combined effect was the best. CLC + APA not only had an effect on the anxiety under the stress state, but also had a regulating effect on the patient's usual anxiety state. On the one hand, local anesthetics before puncture enhanced the confidence of patients to deal with pain and reduced the fear of pain. On the other hand, it was related to the antianxiety effect of APA.

APA can effectively relieve the negative emotions of patients [38, 39], which may be related to acupoint stimulation of the vagus nerve in the auricular concha. Anatomy of the ear shows that the ear nerves are abundant, which is the organ of the vagus nerve outside [35, 40]. There are branches of the vagus nerve in the auricular concha that have a certain regulating effect on the internal organs, especially when the body is under stress. Secondly, there are great auricular nerves, sympathetic nerves, auricular temporal nerves, and occipital nerves, which form a rich neural network and play an important role in regulating the overall mood and function [40]. Stimulating these nerves, long-term adherence by APA will work better for patients with anxiety and other adverse emotions.

### 4.3. Effect of APA Combined with CLC on Comfort

As the highest form of discomfort, pain is the most painful feeling of patients. AVF puncture pain and the adverse emotions caused by the pain can reduce the comfort of patients. Therefore, improving the comfort of patients is an urgent need of patients and is also the goal of nursing work [41]. Strengthening the intervention to mitigate puncture pain of the arteriovenous fistula is of great significance to improve the comfort level of patients.

The results of this study showed that the overall comfort, physiological comfort, psychological comfort, and environmental comfort of the patients were significantly improved. This is mainly due to the reduction of pain. The improvement of environmental comfort is related to the harmonious relationship between nurses and patients in the process of intervention and the improvement of patients' adaptability to the environment with the extension of dialysis time.

In summary, pain management has entered the era of patient participation, multimodal analgesia, and multidisciplinary cooperation. AVF puncture pain intervention in MHD patients has an important impact. APA combined with CLC can effectively relieve the pain of AVF puncture, reduce the negative emotions caused by the pain, promote the comfort of patients, and meet the needs of patients for overall nursing. It is a simple and easy preemptive analgesia intervention method, which reflects the synergistic effect of integrated traditional Chinese and Western medicine and multimodal analgesia and is consistent with the goal of health promotion.

### 4.4. Limitations of the Study

There are some limitations in the application of this study in clinical practice such as higher requirements for nurses' basic theoretical knowledge and skills of APA, differences in nurses' attitudes, knowledge, and pain assessment levels of pain management, application methods of local anesthetics, subjective pain perception, and pain management compliance of patients. These factors have a certain impact on the intervention effect, which needs to be strengthened in practice. In addition, due to the short intervention time, we cannot observe the improvement of prognosis and overall quality of life of patients with AVF puncture pain after long-term intervention, which needs to be further studied and discussed in clinical practice.

### 4.5. Implications for Clinical Nursing

AVF puncture pain needs effective intervention. The combination of APA and CLC can significantly reduce the puncture pain of AVF, even if each is used alone. Nurses can use this study to select appropriate intervention methods to improve AVF puncture pain. In addition, nurses can use APA to manage other symptoms of patients.

## 5. Conclusions

AVF puncture multimodal analgesia based on the concept of advanced analgesia can effectively reduce the pain level of patients with AVF puncture, mitigate patients' anxiety, improve comfort and quality of life, and achieve the purpose of designing the most effective analgesic program for patients and achieve the best results. The results of the study will help highlight the analgesic advantages of Chinese and Western medicine, maximize the analgesic effect, optimize the overall patient comfort, reflect humanized management, and provide a reliable basis for the construction of an AVF puncture pain management model. Moreover, it is of great significance for the development of HD specialty subject, and it is worthy of clinical application and promotion.

## Figures and Tables

**Figure 1:** Study flow diagram.

**Figure 2:** Auricular acupoints for AVF puncture pain.

**Figure 3:** AVF puncture VAS pain score trend within eight weeks in 4 groups. ^*∗*^*P* < 0.05, compared with the control group; ^#^*P* < 0.05, compared with APA and CLC.

**Table 1:** Comparison of general demographic data (*n*, %).

Variable		Control (*n* = 30)	CLC (*n* = 30)	APA (*n* = 30)	APA + CLC (*n* = 30)	*χ* ^*2*^	*P*
Gender	Male	21 (70.00)	20 (66.67)	18 (60.00)	19 (63.33)	0.733	0.086
	Female	9 (30.00)	10 (33.33)	12 (40.00)	11 (36.67)		

Age	18∼44	5 (16.66)	6 (20.00)	4 (13.33)	6 (20.00)	0.818	0.992
	45∼59	14 (46.67)	13 (43.33)	14 (46.67)	12 (40.00)		
	60∼	11 (36.67)	11 (36.67)	12 (40.00)	12 (40.00)		

Marriage	Married	17 (56.67)	18 (60.00)	17 (56.67)	16 (53.33)	1.168	0.978
	Unmarried	7 (23.33)	8 (26.67)	9 (30.00)	8 (26.67)		
	Other	6 (20.00)	4 (13.33)	4 (13.33)	6 (20.00)		

Degree of education	Junior high school and below	9 (30.00)	9 (30.00)	9 (30.00)	8 (26.67)	0.817	0.992
	High school	12 (40.00)	10 (33.33)	11 (36.67)	10 (33.33)		
	College and above	9 (30.00)	11 (36.67)	10 (33.33)	12 (40.00)		

Labor status	Working	17 (56.67)	18 (60.00)	18 (60.00)	19 (63.33)	0.278	0.964
	Workless	13 (43.33)	12 (40.00)	12 (40.00)	11 (36.67)		

Religion	Believer	24 (80.00)	23 (76.67)	23 (76.67)	22 (73.33)	0.373	0.946
	Nonbeliever	6 (20.00)	7 (23.33)	7 (23.33)	8 (26.67)		

Smoking	Smoke	14 (46.67)	13 (43.33)	12 (40.00)	12 (40.00)	0.375	0.935
	Not smoking	16 (53.33)	17 (56.67)	18 (60.00)	18 (60.00)		

Average monthly income (¥)	＜2000	3 (10.00)	4 (13.33)	4 (13.33)	5 (16.67)	1.801	0.937
	2000∼	13 (43.33)	14 (46.67)	16 (53.34)	15 (50.00)		
	≥5000	14 (46.67)	12 (40.00)	10 (33.33)	10 (33.33)		

Payment method	Provincial/municipal MI	13 (43.34)	12 (40.00)	13 (43.34)	12 (40.00)	2.472	0.982
	Resident MI	12 (40.00)	13 (43.34)	12 (40.00)	14 (46.67)		
	NRCMS	4 (13.33)	5 (16.67)	4 (13.33)	4 (13.33)		
	Self-paid	1 (3.33)	0	1 (3.33)	0		

CLC = compound lidocaine cream; APA = auricular point acupressure; MI = medical insurance; NRCMS = new rural cooperative medical system; Resident MI = residents medical insurance.

**Table 2:** Comparison of clinical characteristics of the study sample (*n* = 120, *n*, %).

Variable		Control (*n* = 30)	CLC (*n* = 30)	APA (*n* = 30)	APA + CLC (*n* = 30)	*χ*2	*P*
Primary disease	Hypertension	11 (36.67)	8 (26.67)	10 (33.33)	9 (30.00)	1.498	0.997
	Diabetes	10 (33.33)	12 (40.00)	10 (33.33)	10 (33.33)		
	Nephropathy	8 (26.67)	9 (30.00)	9 (30.00)	9 (30.00)		
	Other	1 (3.33)	1 (3.33)	1 (3.33)	2 (6.67)		

Complications	0	3 (10.00)	4 (13.33)	3 (10.00)	5 (16.67)	1.982	0.992
	1	14 (46.67)	15 (50.00)	16 (53.33)	12 (40.00)		
	2	7 (23.33)	7 (23.33)	6 (20.00)	7 (23.33)		
	≥3	6 (20.00)	4 (13.33)	5 (16.67)	6 (20.00)		

Dialysis duration (years)	＜1	7 (23.33)	7 (23.33)	6 (20.00)	8 (26.67)	0.764	0.993
	1∼2	11 (36.67)	13 (43.33)	12 (40.00)	11 (36.67)		
	≥3	12 (40.00)	10 (33.33)	12 (40.00)	11 (36.67)		

AVF use experiences (month)	＜6	6 (20.00)	8 (26.67)	7 (23.33)	8 (26.67)	1.836	0.994
	6∼	7 (23.33)	8(26.67)	8 (26.67)	9 (30.00)		
	12∼	10 (33.34)	10 (33.34)	9 (30.00)	8 (26.67)		
	≥36	7 (23.33)	4 (13.33)	6 (20.00)	5 (16.67)		

CLC = compound lidocaine cream; APA = auricular point acupressure; PHC = physiological comfort; PSC = psychological comfort; SC = social comfort; EC = environmental comfort.

**Table 3:** Comparison of AVF puncture pain intensity across four groups ($\bar{x}\pm s$).

	Before	1 week after the first intervention	4 weeks after the first intervention	Postintervention
Control	6.69 ± 2.52	6.03 ± 2.12	5.79 ± 2.34	5.48 ± 2.03
CLC	6.27 ± 3.10	4.59 ± 2.00	4.22 ± 1.98	4.03 ± 1.36
APA	6.89 ± 3.01	4.34 ± 2.11	4.57 ± 1.45	4.89 ± 1.27
CLC + APA	6.76 ± 2.32	3.76 ± 1.28	2.46 ± 0.90	1.76 ± 0.08
*F* ^∆^	0.293	7.659	18.454	42.133
*P*	0.83	<0.001^*∗∗∗*^	<0.001^*∗∗∗*^	<0.001^*∗∗∗*^
*η* ^2∆∆^		0.165	0.323	0.521

CLC = compound lidocaine cream; APA = auricular point acupressure; *Before* *=* preintervention; *Post* *=* postintervention. ^*∗*^*P* < 0.05, ^*∗∗*^*P* < 0.01, and ^*∗∗∗*^*P* < 0.001. ^∆^Between 4 group comparisons were made using single factor analysis of variance. ^∆∆^Effect size of 4 group comparisons was made using Cohen's d (*η*^2^).

**Table 4:** Comparison of anxiety before and after intervention ($\bar{x}\pm s$).

	State anxiety				Trait anxiety			
	Before	Postintervention	*t* ^∆∆^	*P*	Before	Postintervention	*t* ^∆∆^	*P*
Control	57.69 ± 13.02	54..42 ± 9.21	5.477	<0.001^*∗∗∗*^	47.24 ± 7.70	44.49 ± 5.15	8.216	<0.001^*∗∗∗*^
CLC	56.22 ± 14.41	50.35 ± 9.80	6.573	<0.001^*∗∗∗*^	48.80 ± 8.51	43.36 ± 8.44	27.386	<0.001^*∗∗∗*^
APA	57.02 ± 13.53	49.47 ± 8.74	8.764	<0.001^*∗∗∗*^	47.60 ± 7.80	39.49 ± 5.87	21.909	<0.001^*∗∗∗*^
CLA + APA	56.76 ± 14.78	41.23 ± 7.58	11.737	<0.001^*∗∗∗*^	49.03 ± 8.66	32.36 ± 5.46	29.212	<0.001^*∗∗∗*^
*F* ^∆^	0.057	11.658			0.348	22.233		
*P*	0.982	<0.001^*∗∗∗*^			0.791	<0.001^*∗∗∗*^		
*η* ^2∆∆∆^		0.232				0.365		

CLC = compound lidocaine cream; APA = auricular point acupressure; *Before* *=* preintervention; *Post* *=* postintervention. ^*∗*^*P* < 0.05, ^*∗∗*^*P* < 0.01, and ^*∗∗∗*^*P* < 0.001. ^∆^Between 4 group comparisons were made using single factor analysis of variance. ^∆∆^Within group comparisons were made using paired-samples T test. ^∆∆∆^Effect size of 4 group comparisons was made using Cohen's d (*η*^2^).

**Table 5:** Comparison of comfort before and after intervention ($\bar{x}\pm s$).

		PHC	PSC	SC	EC	Total
Control	Before	15.67 ± 3.86	22.38 ± 4.90	18.44 ± 5.73	13.56 ± 4.47	69.67 ± 8.26
	After	14.46 ± 2.84	23.67 ± 6.35	16.44 ± 5.71	15.56 ± 3.56	68.46 ± 7.89

CLC	Before	16.03 ± 2.36	22.26 ± 2.00	18.19 ± 3.70	13.36 ± 2.94	68.63 ± 7.20
	After	18.68 ± 3.23	25.27 ± 4.34	19.31 ± 3.26	14.27 ± 2.03	71.67 ± 8.89^*∗*Δ^

APA	Before	14.33 ± 4.25	21.12 ± 3.78	17.58 ± 4.75	13.58 ± 2.56	67.99 ± 9.26
	After	22.67 ± 1.86	28.55 ± 4.57	19.40 ± 5.78	15.02 ± 3.36	82.07 ± 10.39^*∗*Δ^

APA + CLC	Before	14.46 ± 4.49	22.30 ± 4.55	17.83 ± 5.76	14.02 ± 5.01	67.59 ± 4.60
	After	29.66 ± 6.80	32.83 ± 7.48	18.77 ± 4.38	16.66 ± 3.12	93.99 ± 7.86^*∗∗*Δ▲^

*F* ^a^	Before	1.493	0.683	0.170	0.154	0.435
	After	73.549	14.450	2.413	3.207	51.308

*P*	Before	0.220	0.564	0.916	0.927	0.728
	After	<0.001^*∗∗∗*^	<0.001^*∗∗∗*^	0.070	0.026^*∗*^	<0.001^*∗∗∗*^

CLC = compound lidocaine cream; APA = auricular point acupressure; PHC = physiological comfort; PSC = psychological comfort; SC = social comfort; EC = environmental comfort. ^*∗*^*P* < 0.05, ^*∗∗*^*P* < 0.01, and ^*∗∗∗*^*P* < 0.001. *Before* represents the preintervention comparison among the 4 groups; *Post* represents the postintervention comparison among the 4 groups; ^Δ^indicates comparison between any two groups by Least Significant Difference; ^▲^compared with APA and CLC by Least Significant Difference pairwise comparison. ^a^Single factor analysis of variance.

**Table 6:** Comparison of BP and HR before and after intervention ($\bar{x}\pm s$).

		HR	Systolic blood pressure	Diastolic blood pressure
Control	Before	91.67 ± 15.34	144.38 ± 14.56	88.47 ± 5.79
	Post	84.46 ± 11.84	146.67 ± 16.54	86.44 ± 5.08

CLC	Before	89.03 ± 13.49	147.26 ± 12.59	88.19 ± 6.44
	Post	78.68 ± 10.23	140.77 ± 14.29	80.31 ± 3.26^*∗*Δ^

APA	Before	90.33 ± 14.25	145.12 ± 13.73	87.58 ± 4.78
	Post	79.67 ± 11.86	139.55 ± 11.36^*∗*Δ^	75.40 ± 5.78^*∗*Δ^

APA + CLC	Before	91.46 ± 16.09	146.33 ± 13.22	86.83 ± 5.44
	Post	77.66 ± 10.80	132.83 ± 10.40^*∗*Δ^	73.77 ± 4.77^*∗*Δ▲^

*F* ^a^	Before	0.201	0.206	0.498
	Post	5.617	5.409	42.067

*P*	Before	0.896	0.850	0.916
	Post	<0.001^*∗∗∗*^	0.002^*∗*^	<0.001^*∗∗∗*^

CLC = compound lidocaine cream; APA = auricular point acupressure; ^*∗*^*P* < 0.05, ^*∗∗*^*P* < 0.01, ^*∗∗∗*^*P* < 0.001. *Before* represents the preintervention comparison among the 4 groups; *Post* represents the postintervention comparison among the 4 groups; ^△^indicates comparison between any two groups by Least Significant Difference; ^▲^compared with APA and CLC by Least Significant Difference pairwise comparison. ^a^Single factor analysis of variance.

## Data Availability

Data are available based on the request to Dr. Xiaohui Liu and approval by the Institutional Review Board of Henan University of Traditional Chinese Medicine.

## References

[1] Gutierrez-Peña M., Zuñiga-Macias L., Marin-Garcia R. (2021). High prevalence of end-stage renal disease of unknown origin in Aguascalientes Mexico: role of the registry of chronic kidney disease and renal biopsy in its approach and future directions. *Clinical Kidney Journal*.

[2] Zhao L., Ren H., Zhang R. (2021). Clinicopathologic features and prognostic factors in older patients with biopsy-proven diabetic nephropathy. *International Urology and Nephrology*.

[3] Adegbola A., Titilope B., Remigus E., Babaniji O. (2020). Burden of end-stage kidney disease in sub-Saharan Africa. *Clinical Nephrology*.

[4] Kaplan A. A. (2017). Peritoneal dialysis or hemodialysis: present and future trends in the United States. *Contributions to Nephrology*.

[5] Group V. A. W. (2006). Clinical practice guidelines for vascular access. *American Journal of Kidney Diseases*.

[6] Vajihe A., Masoumeh B. N., Nouraddine M. S., Fatemeh E., Zahra P. (2017). Comparison of the effects of hegu point ice massage and 2% lidocaine gel on arteriovenous fistula puncture-related pain in hemodialysis patients: a randomized controlled trial. *Journal of Caring*.

[7] Shabandokht-Zarmi H., Bagheri-Nesami M., Shorofi S. A., Mousavinasab S. N. (2017). The effect of self-selected soothing music on fistula puncture-related pain in hemodialysis patients. *Complementary Therapies in Clinical Practice*.

[8] Figueiredo A. E., Viegas A., Monteiro M., Poli-De-Figueiredo C. E. (2009). Research into pain perception with arteriovenous fistula (AVF) cannulation. *Journal of Renal Care*.

[9] Ghoreyshi Z., Amerian M., Amanpour F., Ebrahimi H. (2018). Evaluation and comparison of the effects of Xyla-P cream and cold compress on the pain caused by the cannulation of arteriovenous fistula in hemodialysis patients. *Saudi Journal of Kidney Diseases and Transplantation: An Official Publication of the Saudi Center for Organ Transplantation, Saudi Arabia*.

[10] Burrai F., Lupi R., Luppi M. (2019). Effects of listening to live singing in patients undergoing hemodialysis: a randomized controlled crossover study. *Biological Research for Nursing*.

[11] Lina G. (2014). Effect of puncture-related pain on the quality of life in patients undergoing maintenance hemodialysis through internal arteriovenous fistula. *Zhong nan da xue xue bao Yi xue ban = Journal of Central South University Medical sciences*.

[12] Aihara S., Yamada S., Shichijo S. (2020). Lidocaine‐propitocain cream, a eutectic mixture of local anesthetics, effectively relieves pain associated with vascular access intervention therapy in patients undergoing hemodialysis: a placebo‐controlled, double‐blind, crossover study. *Therapeutic Apheresis and Dialysis*.

[13] Datema J., Veldhuis J., Bekhof J. (2019). Lidocaine spray as a local analgesic for intravenous cannulation: a randomized clinical trial. *European Journal of Emergency Medicine*.

[14] Mansori K., Soltani-Kermanshahi M. (2020). The effects of eugenol nanoemulsion on pain caused by arteriovenous fistula cannulation in hemodialysis patients: a randomized double-blinded controlled cross-over trial. *Complementary Therapies in Medicine*.

[15] Mahboubi M. (2019). Therapeutic and health benefits of Rose fixed oil (Rowghan-E-Gol). *Traditional and Integrative Medicine*.

[16] Zhou X., Wu Q., Wang Y (2020). Moxibustion as an adjuvant therapy for chronic kidney disease: a systematic review and meta-analysis of 23 randomized controlled trials. *Evidence-Based Complementary and Alternative Medicine: ECAM*.

[17] Akrami R., Hashempur M. H., Tavakoli A (2016). Effects of fumaria parviflora l on uremic pruritus in hemodialysis patients: a randomized, double-blind, placebo-controlled trial. *Jundishapur Journal of Natural Pharmaceutical Products*.

[18] Kaplan Serin E., Ovayolu N., Ovayolu Ö. (2020). The effect of progressive relaxation exercises on pain, fatigue, and quality of life in dialysis patients. *Holistic Nursing Practice*.

[19] Driscoll M. A., Kerns R. D. (2016). Integrated, team-based chronic pain management: bridges from theory and research to high quality patient care. *Advances in Experimental Medicine and Biology*.

[20] Jaime B., Long K., Bevil D., Giles L. (2019). Preemptive analgesia in minimally invasive gynecologic surgery - sciencedirect. *Journal of Minimally Invasive Gynecology*.

[21] Chao H., Yeh L.-C., Chien Yi, Chien C., Dianxu R. (2015). Auricular point acupressure as an adjunct analgesic treatment for cancer patients: a feasibility study. *Pain Management Nursing*.

[22] Yeh C. H., Chien L. C., Lin W. C., Bovbjerg D. H., van Londen G. J. (2016). Pilot randomized controlled trial of auricular point acupressure to manage symptom clusters of pain, fatigue, and disturbed sleep in breast cancer patients. *Cancer Nursing*.

[23] Wirz-Ridolfi A. (2019). The history of ear acupuncture and ear cartography: why precise mapping of auricular points is important. *Medical Acupuncture*.

[24] Yeh C. H., Caswell K., Pandiri S (2020). Dynamic brain activity following auricular point acupressure in chemotherapy-induced neuropathy: a pilot longitudinal functional magnetic resonance imaging study. *Global Advances in Health and Medicine*.

[25] Lee S., Park H. (2018). Effects of auricular acupressure on pain and disability in adults with chronic neck pain. *Applied Nursing Research*.

[26] Yeh C. H., Chien L. C., Balaban D. (2013). A randomized clinical trial of auricular point acupressure for chronic low back pain: a feasibility study. *Evidence-Based Complementary and Alternative Medicine*.

[27] Zhong Q., Wang D., Bai Y.-m., Du S.-z., Song Y.-l., Zhu J. (2019). Effectiveness of auricular acupressure for acute postoperative pain after surgery: a systematic review and meta-analysis. *Chinese Journal of Integrative Medicine*.

[28] Roque M. R., Kakuda S. A. K. (2016). Effects of auriculotherapy on labour pain: a randomized clinical trial. *Revista Da Escola De Enfermagem Da U S P*.

[29] Liu G.-m., Lin R.-y., Lu X.-y., Huang C.-x. (2019). Auricular point sticking for relieving pain in arteriovenous fistula puncture. *Journal of Acupuncture and Tuina Science*.

[30] WHO (1990). *WH: Report on the Working Group on Auricular Acupuncture Nomenclature*.

[31] Huang L. (2005). *Auricular Treatment Medicine: Science and Technology Literature*.

[32] Xi L., Cao F., Xiong W., He F., Zhang L. (2014). The impact of allergic rhinitis on state-trait anxiety. *Zhonghua Er Bi Yan Hou Tou Jing Wai Ke Za Zhi*.

[33] Sanem G., Cimen E., Ouz A., Gokcen G., Sertac C. (2020). Listening to music during arteriovenous fistula surgery alleviates anxiety: a randomized single-blind clinical trial. *World Journal of Transplantation*.

[34] Ting-Lu Z., Cheng-Mei Y. (2011). Study on development and reliability & validity of maintenance hemodialysis patients comfort scale. *Nursing Journal of Chinese People’s Liberation Army*.

[35] Hou P.-W., Hsu H.-C., Lin Y.-W., Tang N.-Y., Cheng C.-Y., Hsieh C.-L. (2015). The history, mechanism, and clinical application of auricular therapy in traditional Chinese medicine. *Evidence-based Complementary and Alternative Medicine*.

[36] Aglio L. S., Abd-El-Barr M. M., Orhurhu V. (2018). Preemptive analgesia for postoperative pain relief in thoracolumbosacral spine operations: a double-blind, placebo-controlled randomized trial. *Journal of Neurosurgery: Spine*.

[37] Kopple J. D., Shapiro B. B., Feroze U (2017). Hemodialysis treatment engenders anxiety and emotional distress. *Clinical Nephrology*.

[38] Kao C. L., Chen C. H., Lin W. Y., Chiao Y. C., Hsieh C. L. (2012). Effect of auricular acupressure on peri- and early postmenopausal women with anxiety: a double-blinded, randomized, and controlled pilot study. *Evidence-based Complementary and Alternative Medicine: eCAM*.

[39] Olshan-Perlmutter M., Carter K., Marx J. (2019). Auricular acupressure reduces anxiety and burnout in behavioral healthcare. *Applied Nursing Research*.

[40] Mercante B., Ginatempo F., Manca A., Melis F., Enrico P., Deriu F. (2018). Anatomo-physiologic basis for auricular stimulation. *Medical Acupuncture*.

[41] Melo G. A. A., Aguiar L. L., Silva R. A., Quirino G. d. S., Pinheiro A. K. B., Caetano J. Á. (2019). Factors related to impaired comfort in chronic kidney disease patients on hemodialysis. *Revista brasileira de enfermagem*.

